The article "Field screening of diverse wheat germplasm for determining their adaptability to semi-arid climatic conditions" was retracted in 2022. Reasons: compromised peer review; a conflict of interest; concerns about the authorship.

# Field screening of diverse wheat germplasm for determining their adaptability to semi-arid climatic conditions

**DOI:** 10.1371/journal.pone.0265344

**Published:** 2022-03-18

**Authors:** Shahzadi Mahpara, Muhammad Shafqat Bashir, Rehmat Ullah, Muhammad Bilal, Salma Kausar, Muhammad Imran Latif, Muhammad Arif, Imran Akhtar, Marian Brestic, Ali Tan Kee Zuan, Ehab A. A. Salama, Abdulrahman Al-Hashimi, Alanoud Alfagham

**Affiliations:** 1 Department of Plant Breeding and Genetics, Faculty of Agricultural Sciences, Ghazi University Dera Ghazi Khan, Dera Ghazi Khan, Pakistan; 2 Soil and Water Testing Laboratory for Research, Dera Ghazi Khan, Punjab, Pakistan; 3 Senior Scientist (Agri Chemistry), Soil and Water Testing Laboratory, Lodhran, Pakistan; 4 Scientific Officer, Soil and Water Testing Laboratory, Narowal, Pakistan; 5 Scientific Officer (Lab), Soil and Water Testing Laboratory, Layyah, Pakistan; 6 Senior scientist (Ento), Regional Agriculture Research Institute, Bahawalpur, Pakistan; 7 Department of Plant Physiology, Slovak University of Agriculture, Nitra, Slovakia; 8 Department of Botany and Plant Physiology, Czech University of Life Sciences, Prague, Czechia; 9 Department of Land Management, Faculty of Agriculture, Universiti Putra Malaysia, Selangor, Malaysia; 10 Agricultural Botany Department, Faculty of Agriculture Saba Basha, Alexandria University, Alexandria, Egypt; 11 Department of Botany and Microbiology, College of Science, King Saud University, Riyadh, Saudi Arabia; Harran Üniversitesi: Harran Universitesi, TURKEY

## Abstract

Wheat (*Triticum aestivum* L.) is an important staple food crop for one third of global population and important crop for securing future food security. Rapid changes in the climate on global scale could be a threat for future food security. This situation urges plant breeders to explore the genetic potential of existing wheat germplasm. This study screened forty diverse wheat genotypes for their yield under two different agroclimatic conditions, i.e., Layyah and Dera Ghazi Khan, Pakistan. Data relating to plant height, peduncle length, flag leaf area, spike length, number of spikelets, number of grains per spike, thousand grain weight, chlorophyll content and grain yield were recorded. The tested wheat genotypes significantly differed for grain yield and related traits. Grain yield was positively correlated with plant height, spike length, spike number, flag leaf length, number of grains per spike, and 1000-grain weight. Biplot obtained from the cluster analysis by Euclidean method grouped the studied genotypes in 3 different groups. The genotypes exhibited 10.77% variability within quadrants, whereas 72.36% variability was recorded between quadrants according to clustering. Dendrogram grouped the tested genotypes into two main clusters. The main cluster “I” comprised of 2 genotypes, i.e., ‘Seher-2006’ and ‘AS-2002’. The cluster “II” contained 38 genotypes based on Euclidian values. Genotypes within same cluster had smaller D^2^ values compared to those belonging to other clusters. The genetic relationships of genotypes provide useful information for breeding programs. Overall, the results revealed that genotypes ‘Line 9733’, ‘Bhakar-2002’, ‘Line A9’ and ‘SYN-46’ had better yield and yield stability under climatic conditions of southern Punjab. Therefore, these genotypes could be recommended for general cultivation in the study region.

The article "Field screening of diverse wheat germplasm for determining their adaptability to semi-arid climatic conditions" was retracted in 2022. Reasons: compromised peer review; a conflict of interest; concerns about the authorship.

## Introduction

Wheat (*Triticum aestivum* L.) nourishes most of the global population and widely cultivated crop around the world [1, 2]. The most popular wheat growing areas in the world are high and mid lands [3]. Limited plant species currently fulfill the dietary needs of human life. Currently, wheat, maize, rice, and sorghum are regarded as the most important staple crops for the global population [1, 4]. Wheat is the most important crop among these and grown on a wide area and used as staple food for a large portion of global population [5, 6]. The economies of developing countries like Pakistan strongly rely on wheat crop. Almost 20% of global energy and protein intake are provided by wheat crop [7]. Wheat crop contributes 9.6% and 1.9% towards economy and gross domestic product of Pakistan, respectively. Wheat production witnessed a 2.5% increase during 2020 and the total annual production of Pakistan was 24.946 million tones [8].

The productivity of wheat crop is severely affected by various biotic and abiotic stresses [5, 9–11]. Introduction of transgenic cotton in Pakistan has aggravated the situation as the long growth period of cotton overlaps with sowing and harvesting of wheat crop [12–14]. Non-availability of early maturing [3], drought-tolerant and high-yielding genotypes [5, 6], low soil fertility [15], and low moisture availability [16, 17] are the major reasons of low wheat production in Pakistan. However, a 60% increase in wheat production is needed by 2050 to feed the rapidly growing population of the world [18]. The production could by increased either by increasing area under cultivation or through increasing per unit yield. The rapid urbanization would not allow increase in the area under production; therefore, increasing yield per unit area would be the only option to augment wheat production in the country [18]. Therefore, yield capacity of existing wheat genotypes should be exploited to fulfill the future wheat demands either through selecting the best suited genotypes for regional climatic conditions or through breeding high yielding genotypes. Both these approaches would require screening for existing genotypes to select the best suited ones or candidate parents for breeding purposes.

The article "Field screening of diverse wheat germplasm for determining their adaptability to semi-arid climatic conditions" was retracted in 2022. Reasons: compromised peer review; a conflict of interest; concerns about the authorship.

The outbreaks of new disease and pests and rapid climate change exert negative impacts on grain yield of wheat crop. Drought stress is one of the mainly abiotic stresses negatively affecting the productivity of wheat and regional and landscape scales [19–21]. A significant decline in the yield [21–23] and related traits of wheat crop has been reported due to drought stress at different phenological stages [11, 24, 25]. However, the extent of yield reduction depends on the phenological stage of wheat crop and reproductive stage is regarded as the most crucial stage where optimum moisture supply is mandatory for higher yield [5, 11, 24]. Drought stress significantly reduces seed germination and plant development [5, 6], flag leaf area, and grain yield [10, 26, 27]. Nevertheless, membrane integrity, pigment content, photosynthetic activity, gas exchange, and cell elongation are also hampered by drought stress [28–30]. Heat stress is another abiotic stress experienced due to ongoing climatic changes and a significant decline in wheat yield is noted due to sudden heat waves [31, 32]. High temperature of heat stress reduces wheat yield by 23%; thus, heat tolerant genotypes should be developed to cope the expected changes in the climate of different regions [33, 34].

Grain yield is a complex trait and driven by several factors of which genotype by environment interactions are considered the most important [30, 35]. Therefore, genotype by environment interaction is widely studied to select the best suited genotypes from the existing ones for specific environmental conditions. Genotypic, phenotypic and grain yield correlations are frequently used to select superior genotypes [36, 37]. Genetic variability and interrelationships between agronomic characteristics in wheat genotypes have shown that grain yield is significantly correlated with all characteristics except plant height [38–40].

Genotype selection should be made for specific set of environmental conditions as genotypes responds differently to varying environments [41]. Environmental conditions under which a genotype is grown strongly affect the growth and yield. Therefore, screening a pool of genotypes for a particular environment will lead to distinct yield rankings [35].

Wheat genotypes with a large genetic base would perform better under different environmental conditions. It is believed that natural and human selection breeding methods have been improved after the first cultivation of wheat. Abiotic stresses significantly affect grain yield; therefore, it is possible to make a wise selection of genotypes for hybridization programs [42, 43]. Correlation and path analysis showed that number of tillers per plant and spikelets per spike had positive direct correlation with grain yield [44, 45]. Therefore, genotypes should be screened with a particular objective. The southern Punjab province of Pakistan has semi-arid to arid-climate and wheat crop often suffers from low moisture availability. Nevertheless, the introduction of transgenic cotton in the cotton-wheat cropping system of the province has initiated several conflicts. Therefore, selection of the best suited genotypes for the region is immediately needed to select the best suited ones for current cultivation and future breeding programs.

The article "Field screening of diverse wheat germplasm for determining their adaptability to semi-arid climatic conditions" was retracted in 2022. Reasons: compromised peer review; a conflict of interest; concerns about the authorship.

Therefore, the current field study was designed to investigate the yield stability of early maturing bread wheat genotypes in three different districts of southern Punjab, i.e., Layyah, Muzafargarh and Dera Ghazi Khan. Selection of the genotypes with high yield capacity and their recommendation for general cultivation in these districts was the major objective of the current study. It was hypothesized that the teste genotypes will significantly differ for yield under the climatic conditions of the studied area. The study will help to select the best suited genotypes for the region.

## Materials and methods

### Experimental site

Three experiments were conducted at three different locations in southern Punjab, Pakistan during wheat growing season of 2019–2020. The experiments were simultaneously conducted at research area of Ghazi University, Dera Ghazi Khan, (29.962611°N, 70.498066°E), research area of College of Agriculture, Bahauudin Zakariya University, Bahadur Sub-campus Layyah (30.979488°N, 70.964622°E) and farmers’ field at Tehsil Kot Addu, District Muzaffagarh (30.474147°N, 70.956198°E). All the experimental sites have semi-arid climate.

### Experimental design

The experiments were designed according to randomized complete block design with a net plot size of 4 m × 5 m at all locations. Forty (40) different genotypes and lines available from different institutions were used in the study. The names and sources of the genotypes are given in Table 1. The seeds of all genotypes were obtained from the respective institutions for research. All experiments had four replications.

**Table 1:** The names and source of different wheat genotypes used in the current study.

Sr no.	Name	Source	Sr no.	Name	Source
1	AS-2002	AARI	21	Miraj-2008	RARI
2	SYM-42	-	22	Line 9701	CIMMYT
3	Line 9733	CIMMYT	23	Line 9736	CIMMYT
4	Line 9779	CIMMYT	24	J-10	-
5	SYN-46	-	25	731	-
6	SYN-50	-	26	B-14	-
7	SYN-32	-	27	J-3	-
8	SYN-83	-	28	Line A9	-
9	Line 9686	CIMMYT	29	Line KTDH-16	-
10	Line 9664	CIMMYT	30	Line -J3	-
11	Line 9883	CIMMYT	31	Line-34 Chakwal	AARI
12	SYN-31	-	32	Line-J10	-
13	Line 9782	CIMMYT	33	Line KLR16	-
14	Line 9725	CIMMYT	34	Line B17	-
15	FSD-83	AARI	35	Line K65	-
16	Bakhar-2002	AZRI	36	Line-B6	-
17	Ayub-2000	AARI	37	KLR-13	-
18	Line 9786	CIMMYT	38	9734	-
19	Line 9757	CIMMYT	39	SYN-33	-
20	Line 9881	CIMMYT	40	Seher-2006	AARI

AARI = Ayub Agricultural Research Institute, Faisalabad, Pakistan; CIMMYT = International Maize and Wheat Improvement Center; AZRI = Arid Zone Research Institute, Bhakkar, Pakistan; RARI = Regional Agricultural Research Institute, Bahawalpur, Pakistan, - = information not available.

The article "Field screening of diverse wheat germplasm for determining their adaptability to semi-arid climatic conditions" was retracted in 2022. Reasons: compromised peer review; a conflict of interest; concerns about the authorship.

### Crop husbandry

The standard crop husbandry practices recommended for the region were opted at each experimental site. The experimental fields were irrigated before preparing seedbed. The seedbed was prepared by ploughing the field twice followed by planking. Seeds were sown with manual seed drill by keeping row-to-row distance of 25 cm. The seed rate was kept 125 kg ha^-1^. The crop was sown on November 14, 16 and 18 at Dera Ghazi Khan, Layyah and Kot Addu, respectively. The fertilizers were applied at 100:60:60 NPK per hectare by using Urea, Diammonium phosphate and Murat of Potash as sources. Irrigation was done at all critical stages to exclude the impacts of moisture stress. The crop was harvested on 16, 18 and 20 April at Dera Ghazi Khan, Layyah and Kot Addu, respectively.

### Data collection

Data relating to chlorophyll index, grain yield, flag leaf area, number of grains per spike, number of tillers per plant, peduncle length, plant height, spike length, and number of spikelets per spike were recorded. Chlorophyll index (SPAD values) were recorded with a SPAD meter at vegetative stage of the plants. Plant height of 10 randomly selected plants from each replication and averaged. The flag leaves of 10 randomly selected plants from each replication were collected and their leaf area was measured with a digital leaf area meter. Number of tillers on 10 randomly selected plants were carefully counted and averaged. The lengths of 10 randomly spikes and their spikelets were measured and averaged. A 1 square meter area from each replication was harvested manually, sun dried and threshed to get grain yield. Three random samples of 1000 grains from each genotype were weighed and averaged to record 1000-grain weight [5].

### Statistical analysis

The normality in the data was tested to meet the assumption of Analysis of Variance (ANOVA). The differences among locations were tested, which indicated that locations were non-significant. Therefore, data of all locations were pooled and used in the analysis. One-way ANOVA was conducted to infer the differences among different genotypes for growth and yield related traits [46]. Least significant difference test at 5% probability was used to separate the means where ANOVA denoted significant differences. The correlation among growth and yield characteristics was computed [47]. Principal components analysis (PCA) was executed in CANOCO 5.0 for the easier interpretation of the data [48]. The principal components with eigenvalues >1 were selected and used for the interpretation of the results. Minimal dataset used in the statistical analysis is given as S1 Dataset.

The article "Field screening of diverse wheat germplasm for determining their adaptability to semi-arid climatic conditions" was retracted in 2022. Reasons: compromised peer review; a conflict of interest; concerns about the authorship.

## Results and discussion

Different genotypes included in the study significantly differed for growth and yield-related traits, i.e., plant height, peduncle length, number of tillers per plant, leaf area index, chlorophyll index, number of spikelets per spike, number of grains per spike, 1000-grain weight, grain and biological yields and harvest index (Table 2).

**Table 2:** Analysis of variance of different growth and yield-related traits of tested wheat genotypes sown under field conditions in three different districts of south Punjab province, Pakistan.

Source	DF	Sum of squares	Mean squares	F value	P value
Plant height					
Genotypes	39	2413.123	61.875	7.950	**< 0.0001**
**Peduncle length**					
Genotypes	39	2286.636	58.632	22.456	**< 0.0001**
**Number of tillers per plant**					
Genotypes	39	489.601	12.554	8.456	**< 0.0001**
**Leaf area index**					
Genotypes	39	556.706	14.275	8.825	**< 0.0001**
**Chlorophyll index**					
Genotypes	39	1152.526	29.552	10.492	**< 0.0001**
**Spike length**					
Genotypes	39	996.833	25.560	6.229	**< 0.0001**
**Number of spikelets per spike**					
Genotypes	39	1782.024	45.693	52.562	**< 0.0001**
**Number of grains per spike**					
Genotypes	39	953.471	24.448	6.308	**< 0.0001**
**1000-grain weight**					
Genotypes	39	1613.222	41.365	24.115	**< 0.0001**
**Grain yield**					
Genotypes	39	2956952.394	75819.292	11.123	**< 0.0001**
**Biological yield**					
Genotypes	39	4567519.886	117115.895	9.507	**< 0.0001**
**Harvest index**					
Genotypes	39	78.711	2.018	1.781	**0.004**

DF = Degree of freedom, bold values in the p value column denote that the respective trait significantly differed among different wheat genotypes included in the current study.

The highest values of plant height, peduncle length, number of tillers per plant, leaf area index, chlorophyll index, number of spikelets per spike, number of grains per spike, 1000-grain weight, grain and biological yields and harvest index were recorded for the genotypes ‘Line 9733’, ‘Bhakar-2002’, ‘Line A9’ and ‘SYN-46’, while ‘Line B6’, ‘SYN-50’, ‘SYN-31’, ‘Line 9686’, and ‘KLR-13’ resulted in the lowest values of these traits (Table 3). These results indicate that ‘Line 9733’, ‘Bhakar-2002’, ‘Line A9’ and ‘SYN-46’ are better tolerated to study area compared to the rest of the genotypes included in the study.

The article "Field screening of diverse wheat germplasm for determining their adaptability to semi-arid climatic conditions" was retracted in 2022. Reasons: compromised peer review; a conflict of interest; concerns about the authorship.

**Table 3:** Growth and yield-related traits of tested wheat genotypes sown under field conditions in three different districts of south Punjab province, Pakistan.

Genotypes	PH (cm)	PDL	NTPP	LAI	CH	SPL (cm)	SPLPS	NGPS	TGW (g)	GY (kg/ha)	BY (kg/ha)	HI
**Line 9733**	104.53 a	24.36 a	7.95 ab	27.44 a	52.64 a	12.72 ab	20.73 a	34.48 a-c	36.32 a	4462.97 ab	8108.88 ab	55.03 a-c
**Bakhar-2002**	103.75 ab	23.77 ab	7.93 ab	27.18 ab	52.44 ab	12.57 a-c	20.13 a	34.53 a-c	36.56 a	4460.66 ab	8110.44 ab	54.99 a-c
**Line A9**	103.722 a	23.67 ab	8.55 a	27.80 a	52.20 ab	12.66 a-c	20.05 a	35.31 a	36.67 a	4451.02 ab	8094.66 ab	54.98 a-c
**SYN-46**	103.60 ab	23.56 ab	7.67 a-c	26.14 bc	52.58 a	12.95 a	18.67 b	33.91 a-d	35.50 ab	4511.15 a	8187.00 a	55.08 a-c
**J-10**	102.70 a-c	22.85 bc	7.45 a-d	25.87 cd	51.25 a-d	11.91 a-d	19.92 a	34.64 ab	36.45 a	4466.37 ab	8025.77 bc	55.64 a
**B-14**	101.48 b-e	21.66 cd	6.66 c-f	25.74 c-e	51.57 a-c	11.52 a-e	17.93 bc	33.83 a-e	34.60 bc	4341.38 c-h	7933.88 c-h	54.71 a-d
**Line 9786**	100.61 c-f	20.73 d-f	6.49 d-g	25.73 c-f	50.37 c-g	10.85 b-h	17.44 cd	33.66 a-f	34.44 bc	4369.07 c-e	7975.11 c-f	54.78 a-d
**AS-2002**	102.10 a-d	21.98 cd	6.86 b-e	25.61 c-g	50.17 c-i	10.90 b-g	18.46 b	33.21 b-h	34.17 cd	4337.84 c-h	7936.22 c-h	54.66 a-e
**Line B17**	100.48 c-f	20.56 d-g	6.32 e-j	25.23 c-h	51.01 b-e	10.78 c-i	16.74 d-h	32.72 c-k	33.46 c-g	4331.36 c-i	7918.11 d-i	54.70 a-e
**SYN-33**	100.68 c-f	20.83 de	6.38 d-i	24.96 c-j	50.25 c-h	11.00 b-f	17.26 c-e	33.42 b-g	33.60 -f	4292.47 f-j	7863.44 g-l	54.59 b-e
**SYM-42**	100.45 c-f	20.64 d-f	6.44 d-h	25.20 c-h	50.48 c-f	10.53 d-j	17.08 c-f	29.46 pq	33.18 d-h	4360.47 c-f	7978.00 c-f	54.65 b-e
**Line 9779**	99.70 d-f	19.62 e-j	5.96 e-l	24.95 d-j	49.95 d-j	9.26 f-m	16.62 d-h	32.50 d-l	32.81 e-j	4371.40 c-e	7880.22 f-k	55.54 ab
**J-3**	99.08 ef	19.62 e-j	6.56 c-f	24.80 d-k	48.88 g-l	9.16 f-m	17.03 d-g	32.94 b-i	33.61 c-f	4351.08 c-g	7949.55 c-g	54.73 a-d
**FSD-83**	99.54 d-f	19.53 e-k	5.72 f-m	24.90 d-k	49.38 f-k	9.86 e-m	15.96 h-k	32.12 d-n	32.87 e-i	4394.53 bc	8014.77 b-d	54.82 a-d
**Line 9736**	99.07 ef	19.25 f-k	5.72 f-m	24.64 e-l	49.18 f-k	9.97 e-l	16.47 e-i	32.54 d-l	33.18 d-h	4374.35 cd	7985.00 c-e	54.77 a-d
**SYN-83**	99.80 d-f	19.73 e-i	5.43 g-m	24.63 e-l	50.17 c-i	10.14 d-k	16.84 d-g	32.91 b-i	33.05 d-h	4313.71 d-i	7894.66 e-j	54.64 b-e
**Ayub-2000**	99.51 ef	19.60 e-k	5.70 f-m	23.98 i-p	49.72 d-k	10.13 d-k	17.45 cd	33.11 b-i	33.80 c-e	4297.15 e-j	7776.22 l-o	55.33 a-c
**Miraj-2008**	99.35 ef	19.52 e-k	6.22 e-k	24.84 d-k	49.42 f-k	9.38 f-m	16.87 d-g	32.83 b-j	33.63 c-f	4310.53 d-j	7904.55 e-j	54.53 c-e
**Line-J3**	99.55 d-f	19.73 e-i	5.88 e-l	24.32 h-n	49.37 f-k	9.82 e-m	15.96 h-k	32.07 e-n	32.83 e-i	4284.08 f-j	7848.44 g-l	54.58 b-e
**Line 9757**	99.32 ef	19.30 f-k	5.94 e-l	25.05 c-i	49.67 e-k	9.53 f-m	16.38 f-i	32.28 d-m	33.06 d-h	4258.47 ij	7811.88 j-n	54.51 c-e
**Seher-2006**	99.61 d-f	19.86 e-h	5.76 e-m	24.55 f-l	49.82 d-j	9.94 e-l	16.17 g-j	31.93 f-n	32.45 f-k	4256.33 ij	7811.33 j-n	54.49 c-e
**Line 9883**	98.85 f	18.76 h-k	5.29 i-m	24.16 h-o	48.83 g-l	9.13 f-m	15.37 j-n	31.43 h-o	32.17 h-m	4339.50 c-h	7934.33 c-h	54.69 a-e
**Line KLR16**	99.00 ef	18.70 h-k	5.14 k-n	24.33 h-m	49.44 f-k	8.91 i-n	15.63 i-m	31.75 g-n	32.31 g-l	4312.11 d-i	7890.22 e-j	54.65 b-e
**Line 9881**	98.42 f	18.26 ijk	5.20 j-n	24.01 i-p	48.66 i-l	8.74 j-o	15.51 j-n	31.31 i-o	32.07 h-m	4321.20 c-i	7906.55 e-j	54.65 b-e
**Line 9725**	99.03 ef	19.00 h-k	5.35 h-m	24.31 h-n	48.76 h-l	9.14 f-m	14.82 m-o	30.94 k-p	31.76 i-m	4291.64 f-j	7861.22 g-l	54.59 b-e
**Line 9782**	98.64 f	18.55 h-k	5.30 i-m	24.50 g-l	48.83 g-l	8.97 h-n	15.68 i-l	31.63 g-n	32.55 f-k	4268.01 h-j	7826.33 i-m	54.53 c-e
**SYN-32**	99.14 ef	19.11 g-k	5.14 k-n	24.30 h-n	49.20 f-k	9.47 f-m	15.33 j-o	31.32 i-o	32.21 h-m	4235.15 j	7779.66 k-o	54.44 c-f
**Line-34 Chakwal**	99.02 ef	18.43 h-k	5.13 k-n	23.95 i-q	48.88 g-l	8.67 j-o	15.71 i-l	31.57 h-n	32.45 f-k	4279.84 g-j	7845.11 h-l	54.55 b-e
**731**	98.57 f	18.58 h-k	5.71 f-m	23.92 i-q	48.65 i-l	9.06 g-n	15.02 l-o	30.98 k-p	31.67 i-m	4285.73 f-j	7854.44 g-l	54.56 b-e
**Line K65**	98.84 f	18.76 h-k	5.33 h-m	23.14 n-s	48.72 h-l	9.21 f-m	15.12 k-o	31.06 j-p	31.78 i-m	4274.28 h-j	7835.44 h-m	54.55 cde
**Line KTDH-16**	98.47 f	18.45 h-k	5.41 g-m	23.86 j-q	48.55 j-l	9.11 g-m	14.95 l-o	30.46 m-q	31.23 lm	4290.36 f-j	7858.33 g-l	54.59 b-e
**Line 9664**	98.14 f	18.30 i-k	4.83 l-o	23.22 m-s	48.46 j-l	8.70 j-o	14.68 no	30.73 l-p	31.61 j-m	4305.93 d-j	7881.55 f-k	54.63 b-e
**Line 9701**	98.16 f	18.12 k	5.14 k-n	22.65 rs	48.43 j-l	8.01 m-q	14.88 l-o	30.34 n-q	31.14 lm	4320.58 c-i	7906.55 e-j	54.64 b-e
**Line-J10**	98.32 f	18.17 jk	5.13 k-n	23.72 k-r	48.44 j-l	8.50 k-o	15.02 l-o	30.91 k-p	31.42 k-m	4289.11 f-j	7857.66 g-l	54.58 b-e
**9734**	98.16 f	18.14 jk	4.73 m-p	23.47 l-r	48.24 kl	8.24 l-p	14.48 o	30.37 n-q	31.04 m	4280.44 g-j	7841.00 h-l	54.59 b-e
**KLR-13**	94.37 g	14.82 l	3.70 pq	22.94 p-s	46.12 mn	7.21 n-q	11.84 p	29.67 o-q	28.81 n	4134.74 k	7699.66 op	53.71 e-g
**Line 9686**	93.28 g	14.08 lm	4.08 n-q	23.11 o-s	45.25 no	6.50 pq	11.80 p	29.46 pq	28.53 n	4146.70 k	7780.00 k-o	53.31 g
**SYN-31**	95.02 g	14.75 l	3.75 o-q	22.77 q-s	47.33 lm	6.95 oq	11.54 p	29.25 pq	28.26 n	4132.05 k	7658.33 p	53.97 d-g
**Line-B6**	94.81 g	14.63 lm	3.57 q	22.28 s	46.07 mn	6.33 q	12.40 p	28.87 q	29.05 n	4126.90 k	7716.44 n-p	53.49 fg
**SYN-50**	92.60 g	13.18 m	3.55 q	23.25 m-s	44.51 o	6.31 q	11.60 p	29.34 pq	28.20 n	4136.48 k	7734.55 m-p	53.49 fg
**LSD 0.05**	**2.58**	**1.49**	**1.13**	**1.18**	**1.55**	**1.87**	**0.86**	**1.82**	**1.21**	**76.57**	**102.93**	**0.98**

Here, PH = plant height, PDL = Peduncle length, NTPP = number of tillers per plant, LAI = leaf area index, CH = chlorophyll index (SPAD value), SPL = spike length, SPLPS = number of spikelets per spike, NGPS = number of grains per spike, TGW = 1000-grain weight, GY = grain yield, BY = biological yield, HI = harvest index. Means followed by different letters are statistically different (p < 0.05) from each other.

The article "Field screening of diverse wheat germplasm for determining their adaptability to semi-arid climatic conditions" was retracted in 2022. Reasons: compromised peer review; a conflict of interest; concerns about the authorship.

The results of the current study revealed that peduncle length was positively correlated with spike length, flag leaf length, number of grains per spike, 1000-grain weight, and grain yield (Table 4). Grain yield had positive correlations with flag leaf area, plant height, spike length, number of grains per spikes and 1000-grain weight.

**Table 4:** Correlation matrix for different morphophysiological traits of different wheat genotypes used in the study.

	CHL	GY	FLA	NGPS	NTPP	PDL	PH	SPL	SPLPS
**GY**	0.4734**								
**LAI**	0.6798**	0.6362**							
**NGPS**	-0.6939*	0.4678*	0.6842**						
**NTPP**	0.7882**	0.661**	0.8495**	-0.6908**					
**PDL**	-0.8744**	-0.6179**	-0.7587**	-0.7507**	0.8253**				
**PH**	0.7629**	0.5784**	0.6347**	0.5244**	0.8308*	0.7199**			
**SPL**	0.7839**	0.3049*	0.6259**	0.7135**	0.6291**	0.8840*	0.4576*8		
**SPLPS**	0.7837**	0.7525**	0.7619**	0.7746**	0.8256**	0.8231*	0.7346**	-0.6135**	
**TGW**	0.7512**	0.6956**	-0.7796**	-0.8323**	0.7848**	0.913**	0.5913**	0.7914**	-0.9096**

Significant

**≤0.01

*≤0.05; Here CHL = chlorophyll index, GY = grain yield, FLA = flag leaf area, NGPS = number of grains per spike, NTPP = number of tillers per plant, PDL = peduncle length, PH = plant height, SL = spike length, TGW = 1000-grain weight and SPLPS = number of spikelets per spike.

Principal component analysis conducted on the growth and yield related traits of the wheat genotypes included in the study yielded only one principal component with eigenvalue > 1 (Table 5). The first principal component explained 85.70% variability in the data, and it was positively influenced by all of the growth and yield-related traits. Biplot obtained from the cluster analysis grouped the genotypes in to 3 different groups (Fig 1). The first group was influenced by biological and grain yields and harvest index. The second group was influenced by the rest of the studied traits, while third group was not influenced by any of the studied traits (Fig 1).

The article "Field screening of diverse wheat germplasm for determining their adaptability to semi-arid climatic conditions" was retracted in 2022. Reasons: compromised peer review; a conflict of interest; concerns about the authorship.

**Fig 1:** Biplot of first two principal components resulting from the principal component analysis executed on different growth and yield-related traits of forty different wheat genotypes included in the study. Here, PH = plant height, PDL = Peduncle length, NTPP = number of tillers per plant, LAI = leaf area index, CH = chlorophyll index (SPAD value), SPL = spike length, SPLPS = number of spikelets per spike, NGPS = number of grains per spike, TGW = 1000-grain weight, GY = grain yield, BY = biological yield, HI = harvest index.

**Table 5:** Eigenvalues, variability explained and factor loadings of first four principal components obtained as a result of principal component analysis executed on growth and yield related traits of fort different wheat genotypes included in the study.

	PC1	PC2	PC3	PC4
**Eigenvalue**	10.28	0.96	0.25	0.17
**Variability (%)**	85.70	8.05	2.13	1.45
**Cumulative variability %**	85.70	93.75	95.89	97.34
**Factor loadings**				
Plant height	0.96	-0.19	-0.04	-0.11
Peduncle length	0.96	-0.18	-0.06	-0.10
Number of tillers per plant	0.95	-0.08	-0.12	0.05
Leaf area index	0.95	-0.10	-0.14	0.07
Chlorophyll index	0.95	-0.18	-0.01	-0.12
Spike length	0.95	-0.18	-0.04	-0.13
Number of spikeletes per spike	0.97	-0.11	0.09	0.07
Number of grains per spike	0.92	-0.12	0.25	0.20
Thousand grain weight	0.96	-0.11	0.09	0.13
Grain yield	0.85	0.51	-0.02	-0.00
Biological yield	0.81	0.50	-0.23	0.11
Harvest index	0.80	0.49	0.26	-0.17

Results presented in Table 6 indicate descriptive statistics of the measured growth and yield-related attributes of different wheat genotypes included in the study. Plant height varied from 87.8 to 107.53 cm. Peduncle length varied between 12.73 and 26.16 cm with mean value of 19.26 cm. Number of tillers per plant varied between 2.53 and 9.23. Flag leaf area ranged between 21.06 and 28.86 cm^2^. Chlorophyll index varied between 39.86 and 54.86. Spike length raged between 5.23 and 16.71 cm. Number of grains per spike ranged between 22.20 and 36.70 indicating a large variation among the tested genotypes. Grain yield is a complex trait driven by genotype by environmental interactions. One of the significant resources in genetic improvement is selection. Some of the researchers have reported substantial variation among genotypes for grain yield and related traits [49], including number of grains per spike [37], straw yield, weight of 1000 kernels, biological yield and harvest index [50–52].

The article "Field screening of diverse wheat germplasm for determining their adaptability to semi-arid climatic conditions" was retracted in 2022. Reasons: compromised peer review; a conflict of interest; concerns about the authorship.

**Table 6:** Descriptive statistics for different morpho-physiological traits of 40 wheat genotypes included in the study.

Variable	Minimum	Maximum	Mean	Standard deviation
**PH**	87.80	107.53	99.21	3.53
**PDL**	12.73	26.16	19.26	2.74
**NTPP**	2.53	9.23	5.72	1.38
**LAI**	21.06	28.86	24.52	1.52
**CHL**	39.86	54.86	49.29	2.11
**SPL**	5.23	16.70	9.56	2.34
**SPLPS**	11.33	20.83	16.03	2.26
**NGPS**	22.20	36.70	31.89	1.97
**TGW**	27.40	37.66	32.60	2.28
**GY**	4034.66	4634.33	4308.56	111.99

Here CHL = chlorophyll index, GY = grain yield, FLA = flag leaf area, NGPS = number of grains per spike, NTPP = number of tillers per plant, PDL = peduncle length, PH = plant height, SL = spike length, TGW = 1000-grain weight and SPLPS = number of spikelets per spike.

Cluster analysis by Euclidean method grouped the tested wheat genotypes in to 4 quadrants (Fig 2) according to dissimilarity matrices. All the genotypes showed 10.77% variability within quadrant, while 72.36% variability was recorded between quadrants. The genotypes placed in similar quadrant had lesser variability, while genotypes in different quadrants had higher variability. Indirect selection can be applied in the case where the same character is measured on the same genotypes in different environments. The phenotypic association between environments can be used to examine indirect response to selection if there are no associations between error effects between environments [53]. An average environmental coordination process [54] assessed the yield efficiency and stability of genotypes.

**Fig 2:** Dendrogram resulting from the cluster analysis executed on different growth and yield-related traits of forty different wheat genotypes included in the study. The genotype codes are given in Table 1.

The dendrogram obtained from the cluster analysis by Euclidean method grouped the tested wheat genotypes into two main clusters according to dissimilarity matrices. The genotypes were grouped into two major clusters I and II. Main cluster “I” comprised of 2 genotypes, i.e., Seher-2006 and AS-2002, whereas the remaining 28 genotypes were grouped in the cluster “II”. Euclidian distances between pairs of genotypes are widely used as a measure of dissimilarity [55, 56]. The genotypes were divided into two clusters in such a way that all the genotypes within the cluster had smaller D^2^ values among than those belonging to different clusters. Awareness of genetic relationships between genotypes offers valuable knowledge to tackle selective breeding and the control of germplasm capital. The current cluster analysis results are in line with those obtained by [57–59], who reported that agronomic parameters were useful using conventional cluster analysis in the clustering of flax, triticale and barley.

The article "Field screening of diverse wheat germplasm for determining their adaptability to semi-arid climatic conditions" was retracted in 2022. Reasons: compromised peer review; a conflict of interest; concerns about the authorship.

## Conclusion

The tested genotypes exhibited significant variability for yield related traits. The cluster analysis divided the genotypes into two major groups based on dissimilarity matrix. Overall, the results revealed that genotypes ‘Line 9733’, ‘Bhakar-2002’, ‘Line A9’ and ‘SYN-46’ had better yield and yield stability under climatic conditions of Dera Ghazi Khan. Therefore, these genotypes could be recommended for general cultivation in the study region.

## Supporting information

S1 Dataset Minimal dataset of the study used in the statistical analysis. (XLSX)
